This article has been retracted.

# Marathon Runner with Acute Hyponatremia: A Neurological Disorder

**DOI:** 10.1155/2012/342760

**Published:** 2012-05-31

**Authors:** R. Kormann, F. Philippart, S. Hubert, C. Bruel

**Affiliations:** ^1^Internal Medicine, Groupe Hospitalier Paris Saint Joseph, 75014 Paris, France; ^2^Intensive Care Unit, Groupe Hospitalier Paris Saint Joseph, 75014 Paris, France; ^3^Paris Descartes University, 75006 Paris, France

## Abstract

We report the case of an athletic 49-year-old female who has run the 2011 Marathon of Paris and was addressed to the hospital for a confusion. The investigations revealed a cerebral edema complicating a severe hyponatremia secondary to an exercise-associated hyponatremia (EAH). Using 3% hypertonic saline solution, the evolution the patient rapidly improve allowing discharge after 7 days. We then discuss the importance of EAH in long-term efforts.

## 1. Introduction 

Marathons, and more widely long-term efforts attract more and more nonprofessional runners (popular festive events and charity runs). Due to this modification of population behavior, pathologies associated with high-level sport practices tend to take a huger place in emergency clinical practice. Among them, exercise-associated hyponatremia (EAH) is a very important one.

## 2. Case Presentation

We report the case of an athletic 49-year-old female with no medical records who has run the 2011 Marathon of Paris (42.195 Km). In view of the marathon, the patient started to train a few months ahead as per two to three runs weekly. She completed the marathon within 5 h 30, with an average speed of 7.5 Km/h, on a warm day (27 degrees celsius). Along the run, she drunk 4 L of mineral water (5 mg/L NaCl), and had some energy bars at the various feeding stations. Four hours after completion of the marathon, the patient felt dizzy and nauseous, with a strong asthenia and encompassed three vomiting periods associated with disorientation and confusion. She was then admitted to the emergency room 7 hours after the afore-mentioned symptoms occurred.

Upon admission, the patient was conscious but disoriented, clouded, with a Glasgow coma score of 13. She was apyretic and presented no circulatory failure. The neurological examination revealed acute spreadover of osteotendinous reflexes the four limbs, no systematic deficiencies and cutaneous plantar reflexes in flexion, isochoric and reactive pupils. Her body weight was 53.4 Kg (normal average body weight of 50 Kg).

The patient was then transferred to the intensive care unit (ICU) for diagnosis and treatment. Four hours later, the patient had a generalized tonic-clonic seizure that resolved following 1 mg clonazepam IV injection. The cerebral CT-scan showed a diffused supratentorial cerebral oedema (Figure 1). The initial biological parameters were natremia 121 mmol/L, chloremia 88 mmol/L, protidemia 70 g/L, glycemia 8.5 mmol/L, kalemia 3.3 mmol/L, bicarbonates 18 mmol/L, blood urea nitrogen 3.7 mmol/L, creatinemia 68 *μ*mol/L, blood urea nitrogen 2.9 mmol/L, uric acid 214 mmol/L, Glycemia 6.6 mmol/L, calcemia 1.8 mmol/L, phosphorus 0.87 mmol/L, magnesemia 1.04 mmol/L, CPK 14486 UI/L, Hb 10.1 g/dL, platelet count 172 G/L, and leukocytes 11.06 G/L. The calculated osmolality was 260 mosm/kg and the measured osmolality was 246 mosm/kg. Arterial blood gases showed a respiratory alkalosis to compensate an increased plasmatic anion gap metabolic acidosis, with initial blood lactate 10.5 mmol/L. The initial collection of a urine sample showed an urinary osmolality of 489 mosm/L. We report a natriuresis and kaliuresis of 86 and 75 mmol/L, respectively. The measure of the free cortisol was 1250 nmol/L at 8 am, and 1350 nmol/L following the ACTH test, by which therefore eliminate an adrenal origin of hyponatremia.

 The patient was given a calculated bolus of isotonic saline as per the Adrogue formula. As no further clinical improvements followed, with a persistent hyponatremiaof 121 mmol/L, the patient was given a treatment based on 3% hypertonic saline solution. Natremia was recorded and indicated 128 mmol/L and 136 mmol/L at 4 hours and 7 hours after beginning of the treatment, respectively. Despite a rapid correction of natremia abnormalities, biological improvement was associated with the resolution of the neurological perturbations without apparition of new neurological symptoms.

The patient was discharged after 7 days following complete resolution of clinical and biological disorders.

## 3. Discussion

The clinical and biological context is a physical exercise-associated hyponatremia(EAH) as defined by a plasmatic sodium concentration below 135 mmol/L 24 h following a prolonged physical activity [1, 2]. Marathons attract plenty of nonprofessional runners like our patient who ran her first marathon at the age of 49. Risk factors in favor of EAH occurrence can be merged into two groups: (i) runner condition-associated factor (female, low body weight, lack of training, slow runner, excessive drinking consumption during the run, and NSAIDS consumption); (ii) environment-related factors (prolonged physical activity of over 4 h, warm air temperature, and drinks availability along the run [3]).

This syndrome, first described in 1981 [1], is closely related to an evolution in high-level sport practices (marathon; triathlon) and the concept of abundant hydration during the activity in order to reduce dehydratation and hypernatremiarisks [4]: an overdrinking consumption during and after the run, and the related occurrence of a syndrome of inappropriate secretion of antidiuretic hormone (SIADH). The excessive drinking consumption during activity is the primary and critical risk factor associated to EAH occurrence [4, 5]. Then, it has been shown that the risk to develop an EAH is correlated to an increase of body weight during the physical activity as observed in the present patient (+3,4 Kg). There are no indications of a thirst deregulation among runner, as thirst is a late adaptation mechanism in this particular regulation system [6]. Despite this, the hyperhydratation during activity on its own cannot resume hyponatremia. The kidneys can excrete 750 to 1500 mL/h of water in normal physiological conditions [7]. ADH is a hormone secreted by the hypothalamus and is subject to stimulation upon low charges (1-2%) in the plasmatic osmolality [8]. In addition to the osmotic stimulation, other mechanisms inducing the central production of ADH have been described: nausea, vomiting organic stress, pain and endorphins, volemic status, central temperature increase, or hypoxia [2, 4, 6–9]. The excess of ADH production is responsible for potentially serious hyponatremiaas described by Siegel et al. [10] and recognized as a key factor for the EAH occurrence [2, 4, 7, 9, 10]. Moreover, It has been suggested that cytokines release (IL6) could also be involved in the nonosmotic stimulation of ADH [7, 9]. A rapid decrease of natremia (<128 mmol/L) is correlated with the emergence of serious clinical alterations, notably neurological disorders following brain swelling [3], as described in the present patient. Patients associated with symptomatic EAH and subsequent serious neurological (confusion, vigilance disorders, coma, and tonic-clonic seizures) or pulmonary (acute respiratory failure) disorders should imperatively be transferred to ICU with a repeated surveillance as the natremia. Acute hyponatremia treatment can benefit of a novel concept associated with a remarkable therapeutic efficiency [2, 4, 7, 9, 10]. Treatment of serious EAH conditions involve the administration of a 3% hypertonic saline solution at 1 mL/kg/h, that is subsequently adjusted following natremia status. Increases of natremia to 1 mmol/L/h during the first 6 h, 9 mmol/L during the first 24 h, and 18 mmol/L during the first 48 h are accepted. Ideally, natremia should not evolve over 20–25 mmol/L during the first 48 h [5, 10]. The isotonic saline solution appears inefficient for the treatment of EAH as described in a previous study [4] and as observed in the present case, in which no noticeable positive biological response was detected following initial administration of saline. 

The EAH prevention relies on information regarding hyperhydratation risks during the run and the necessity to control water supplies in a range of 400–700 mL/h, depending on body weight and weather conditions [5]. Beltrami has described the historical link between overdrinking during a prolonged and intensive sport activity and the occurrence of hyponatremia. This overdrinking behavior seems to be supported by sport drinks selling companies. Moreover, these sport drinks (enriched solutions with mineral salts and ions, slightly less hypotonic than mineral water) do not prevent EAH, neither is the sodium supplier by systematic per os intake [3].

## 4. Conclusion

In summary, EAH is associated to a SIADH which the severity is as high as the hydric supply during and after the physical activity, occurring during or in the few hours following the activity. It could sometimes evolve as critical emergency situation with signs of neurological disorders, and the only efficient treatment consists of the administration of hypertonic saline solution. The prevention strategy consists in informing runners on good hydration practices during the run and the hyperhydratation-associated risks.

## Figures and Tables

**Figure 1:** Noninjected CT-scan realized on the day of admission.
